# Ruscogenin Ameliorated Sjögren's Syndrome by Inhibiting NLRP3 Inflammasome Activation

**DOI:** 10.1155/2022/6425121

**Published:** 2022-06-28

**Authors:** Jing He, Yue Wang, Lei Xu, Changsong Xu, Yamei Zhu, Meimei Xu, Yueyue Chen, Liang Guo, Wei Hu, Dake Xu, Rongyue Jing, Bo Xu

**Affiliations:** ^1^Department of Immunology and Rheumatology, Third Affiliated Hospital of Nanjing University of Traditional Chinese Medicine, Nanjing, Jiangsu, China; ^2^Department of First Clinical Medical College, Nanjing University of Traditional Chinese Medicine, Nanjing, Jiangsu, China

## Abstract

This article investigated the role and the specific mechanism of Ruscogenin in Sjögren's syndrome (SS). NOD/ShiLtJ mice were treated with Ruscogenin, and acinar cells isolated from submandibular glands were treated with TNF-*α*, Ruscogenin and transfected with NLRP3 overexpression plasmid. Salivary flow rate (SFR) was measured at weeks 11, 13, 15, 17, and 20. Histological analysis of the submandibular glands was conducted by hematoxylin-eosin staining assay. IL-6, IL-17, TNF-*α*, and IL-1*β* mRNA expression was detected through qRT-PCR. AQP 5, AQP 4, P2X7R, NLRP3, caspase 1, IL-1*β*, Bax, and Bcl-2 protein levels were tested by western blot. Cell apoptosis was assessed through acridine orange and propidium iodide (AO/PI) staining assay and flow cytometry assay. Ruscogenin ameliorated the SFR and submandibular gland inflammation of NOD/ShiLtJ mice. Ruscogenin promoted the preservation of acinar cells and suppressed inflammation-related factors (P2X7R, NLRP3, caspase 1, and IL-1*β*) in submandibular gland tissues of NOD/ShiLtJ mice. Ruscogenin inhibited acinar cell apoptosis in NOD/ShiLtJ mice and reversed TNF-*α*-induced apoptosis and inflammation of acinar cells. NLRP3 overexpression reversed the repressive effect of Ruscogenin on TNF-*α*-induced inflammation and apoptosis of acinar cells. Ruscogenin ameliorated SS by inhibiting NLRP3 inflammasome activation.

## 1. Introduction

As the prevalence ranges from 0.1% to 0.72% among the population around the world with a female preponderance (The ratio of female to male is 9 : 1), Sjögren's syndrome (SS), usually classified as the primary (occurs by itself) and the secondary (relates to other autoimmune diseases like rheumatoid arthritis or lupus), is an autoimmune disorder distinguished by exocrine gland (typically lachrymal and salivary glands) dysfunction owing to infiltration of lymphocytes, leading to excessive dry eyes (keratoconjunctivitis sicca) and dry mouth (xerostomia) [1–4]. In general, the immune system targets epithelial tissues, then infiltrates with them with lymphocytes, and finally generates autoantibodies against antigens of glands [2]. What's worse, SS is able to develop from disease limited to the exocrine glands to diverse extraglandular manifestations including chronic fatigue, arthralgias, nonerosive polyarthritis, vasculitis, and even lymphoma [5, 6]. And with the slow progression of SS, patients with the disease are more likely to perform clinical symptoms years after the disease onset [7]. Without effective treatment of SS, the current SS interventions such as saliva substitutes and medications (cevimeline, pilocarpine, etc.) are symptomatic-based, which can only offer a temporary relief of dryness severity and complications, resulting in economic, physical, and mental burdens on patients with SS [2, 8, 9]. Hence, it is of urgent significance to search for novel agents with favorable efficacy for SS therapy.

Although the causes of SS remain largely unknown, the inflammation is a well-defined condition among all cases with SS, which can partly attribute to aberrant innate and adaptive immune reactions implicated in pathogenesis of SS [10–12]. Besides, the hyposalivation and glandular destruction induced by chronic inflammation during SS are considered to be associated with the injury of acinar cells [13, 14]. Inflammasomes are a class of multimeric protein complexes fulfilling a critical function on an innate immune system, the activation of which promotes maturation and secretion of pro-inflammatory cytokines and modulates caspase-1 for further inflammatory events and apoptosis [11, 15]. Former studies have shown that nucleotide binding oligomerization domain-like receptor 3 (NLRP3) inflammasome is activated in patients with SS [11], which suggested that NLRP3 inflammasome may act as a therapeutic target for SS management.

Ophiopogon japonicas is a common traditional Chinese herbal medicine mainly consisting of polysaccharides, saponins, and homoisoflavonoidal compounds, whose clinical efficacy like antithrombotic activity and anti-inflammatory property has been validated by scientific evidence [16–18]. Moreover, Ophiopogon japonicas is theoretically regarded to realize an effect of “moisturize dryness and facilitate to produce body fluid” and has been utilized in the treatment of xerosis-related dysfunction with traditional Chinese medicine for a long time [16]. As a major bioactive steroid sapogenin isolated from Ophiopogon japonicas, Ruscogenin has been extensively applied in the treatment for chronic inflammation and cardiovascular diseases [18, 19]. Additionally, its anti-inflammatory and antithrombotic activities greatly contribute to the improvement of mouse neutrophil activation, cerebral ischemic injury, and pulmonary arterial hypertension [20–22]. Nevertheless, the effects of Ruscogenin on SS are largely unknown. Previous studies have reported that Ruscogenin can mitigate blood-brain barrier dysfunction induced by cerebral ischemia through the inhibition of the MAPK pathway and TXNIP/NLRP3 inflammasome [23], and MDG-1 (also named Ophiopogon japonicas polysaccharides), another component of Ophiopogon japonicas, has been confirmed to alleviate symptoms of SS [16]. Those findings suggest that Ruscogenin may regulate NLRP3 inflammasome to impact upon SS. Therefore, this study attempted to explore the role of Ruscogenin in SS as well as the specific mechanisms involved through in vivo and in vitro experiments on a basis of NLRP3 inflammasome.

## 2. Materials and Methods

### 2.1. Animals

Female NOD/ShiLtJ mice aged 8 weeks [2] (*n* = 40, weighed 18–22 g) were bought from The Jackson Laboratory (Bar Harbor, ME, USA), while female BALB/c mice (*n* = 10, aged 8 weeks, weighed 18–22 g) were obtained from Beijing Vital River Laboratory Animal Technology Co., Ltd. (Beijing, China) as a control. All the mice were allowed free access to food and water, and maintained under specific pathogen-free conditions as well as a relative humidity of 50 ± 20%, an ambient temperature of 22 ± 3°C, and a constant cycle of 12-h light/dark.

### 2.2. Drug Preparation

Extracted from the tuber of Ophiopogon japonicus, Ruscogenin was purified by successive chromatographic steps until the purity of the sample analyzed using high-performance liquid chromatography-evaporative light scattering detection (HPLC-ELSD) reached 98.6% [23].

### 2.3. Drug Treatment

Ruscogenin was dissolved in sterile phosphate buffer saline (PBS; C0221A, Beyotime Biotechnology, Shanghai, China). Treatments were administered orally every day, lasting for 9 weeks. NOD/ShiLtJ mice were randomized into four groups (*n* = 10 per group). The NOD/ShiLtJ group was normally reared without any treatment; the vehicle group was administered vehicle (an equal volume of sterile PBS); the Ruscogenin 0.3 group was treated with Ruscogenin at 0.3 mg/kg body weight; and the Ruscogenin 1 group was treated with Ruscogenin at 1 mg/kg body weight.

### 2.4. Measurement of Salivary Flow Rate (SFR)

NOD/ShiLtJ mice were anesthetized by isoflurane (2%) inhalation, following which they were injected intraperitoneally with pilocarpine (C11H16N2O2; 1538505, Sigma-Aldrich, St. Louis, MO, USA) at a concentration of 5 mg/kg for the stimulation of salivary secretion. Saliva was then collected for 7 min using a 200 *μ*L pipette (SE4-200XLS+, Mettler Toledo, Zurich, Switzerland, https://www.mt.com/cn/zh/home.html), which was adopted to evaluate the total volume. SFR is performed in microliters per gram of body weight per min (*μ*L/gm/min).

### 2.5. Histological Analysis

Histological analysis of the submandibular gland was performed at week 20 after NOD/ShiLtJ mice were sacrificed via euthanasia using 100 mg/kg ketamine in combination with 5 mg/kg xylazine. The submandibular glands removed from NOD/ShiLtJ mice were fixed in 10% neutral buffered formalin (G2161, Beijing Solarbio Science & Technology Co., Ltd., Beijing, China) for 24 h, and dehydrated and embedded in wax. Serial sections of the tissues at a thickness of 5 *µ*m were taken through an automated microtome (Leica RM2235, Leica Microsystems, Wetzlar, Hesse-Darmstadt, Germany, https://www.leica-microsystems.com.cn/cn/). Hematoxylin-Eosin (HE) Staining Kit (G1120, Beijing Solarbio Science & Technology Co., Ltd., China) was utilized for tissue stain. In brief, after deparaffinization in xylene (C8H10, ≥75.0%; 214736, Sigma-Aldrich, USA) twice for 5 min and hydration in 100% ethanol for 5 min, 95% ethanol for 2 min, 80% ethanol for 2 min, and 70% ethanol for 2 min, as well as distilled water for 2 min, the sections were immersed in hematoxylin solution for 5 min and rinsed by water. Sections were then differentiated by differentiation liquid for 30 s, followed by immersion in water for 15 min. Subsequently, sections were immersed in 0.6% ammonia water for 15 min to make the nucleus return back to blue and washed with water. Next, eosin solution was applied to stain sections for 2 min and rinsed with water. Sections were quickly dehydrated in 75% ethanol for 3 s, 85% ethanol for 3 s, 95% ethanol for 3 s, 100% ethanol for 3 s, and 100% ethanol for 1 min, made to be transparent in phenol (C6H6O, ≥99.0%; P1037, Sigma-Aldrich, USA) and xylene (1 : 3) for 1 min and xylene twice for 1 min, and eventually mounted in a resinous medium. Specimens were observed under a microscope (magnification: ×100; Leica DM IL LED, Leica Microsystems, Germany).

### 2.6. Quantitative Reverse Transcription-Polymerase Chain Reaction (qRT-PCR)

Tissues were ground in advance through a D-500 homogenizer (Wiggens, Straubenhardt, Germany, http://www.wiggens.com/), following which total mRNA of tissues was extracted using RNAiso Plus (Trizol) (9109, Takara Biomedical Technology Co., Ltd., Beijing, China). Then, the PrimeScript™ RT Reagent Kit with gDNA Eraser (Perfect Real Time) (RR047A, Takara Biomedical Technology Co., Ltd., China) was employed to synthesize cDNA during reverse transcription. Next, cDNA was amplified in Applied Biosystems 7300 Real-Time PCR System (ABI, Thermo Fisher Scientific, USA) under a condition including predenaturation at 95°C for 30 s, 40 thermal cycles of 95°C for 5 s and 60°C for 31 s, which was traced by TB Green® Premix Ex Taq™ II (Tli RNaseH Plus) (RR820Q, Takara Biomedical Technology Co., Ltd., China). The primer sequences (Guangzhou RiboBio Co., Ltd., Guangzhou, China) are presented in Table 1. Glyceraldehyde-3-phosphate dehydrogenase (GAPDH) is the endogenous control, and data were calculated via the 2-ΔΔCT relative quantification method [24].

### 2.7. Isolation of Acinar Cells in Submandibular Gland

Submandibular glands were quickly removed and immediately transferred to ice-cold Roswell Park Memorial Institute (RPMI)-1640 Medium (E600028, Sangon Biotech Co., Ltd., Shanghai, China) enriched with 10% fetal bovine serum (FBS; 11011–8611, Beijing Solarbio Science & Technology Co., Ltd., China). Then, the tissues were minced into small pieces, followed by digestion in 2.5 ml RPMI-1640 medium supplemented with 0.1 g/L soybean trypsin inhibitor (17075029, Thermo Fisher Scientific, Waltham, MA, USA), 10% FBS, and 100 U/ml Collagenase IV (17104019, Thermo Fisher Scientific, USA) in a shaking water bath at a speed of 120 cycles/min for 10 min at 37°C. At last, the mixture was dispersed using a plastic pipette and filtered through a 150-mesh nylon net. The acinar cells extracted from submandibular glands of female BALB/c mice were taken as a control.

### 2.8. Acridine Orange and Propidium Iodide (AO/PI) Staining Assay

AO/PI Staining Apoptosis Detection Kit (BB-4142-1, Bestbio, Shanghai, China, http://www.bestbio.com.cn/) was utilized to test cell apoptosis. Reagent C (100 *μ*L) was mixed with sterile deionized water (900 *μ*L) to make staining binding buffer. Cells (1 × 10^6^) were washed twice with PBS and resuspended in 500 *μ*L staining binding buffer. AO staining solution (5 *μ*L) and PI staining solution (5 *μ*L) were added to cells in turn and mixed gently, following which cells were incubated at 4°C in a dark room for 20 min. Cells were then rinsed by PBS and observed using the Leica DM IL LED microscope (magnification: ×200).

### 2.9. Acinar Cell Treatment

Normal acinar cells were pretreated with Ruscogenin (0.1, 1, 10 *µ*M) for 24 h [23], which is followed by the treatment of TNF-*α* (10 ng/mL; Z02774, Genscript, Nanjing, China, https://www.genscript.com.cn/) for 8 h [25].

### 2.10. Flow Cytometry Assay

Cell apoptosis was detected by Annexin V-FITC/PI Apoptosis Detection Kit (E606336, Sangon Biotech Co., Ltd., China). Cells were rinsed with PBS and suspended in 1 × binding buffer (195 *μ*L) at a density of 2 × 10^5^ cells/mL. Next, 5 *μ*L Annexin V-FITC was added and mixed well in a dark room, followed by culture for 15 min at room temperature. Then, cells were washed by 1 × binding buffer (200 *μ*L) and centrifuged for 5 min at 1000 rpm. As the supernatant was removed, cells were resuspended in 1 × binding buffer (190 *μ*L) with 10 *μ*L PI. A CytoFLEX S flow cytometer (Beckman Coulter, Inc., Brea, CA, USA) was adopted for cell apoptosis analysis.

### 2.11. Cell Transfection

The overexpression vector (pcDNA3.1/+vector; V79020, Invitrogen, Thermo Fisher Scientific, USA) carrying NLRP3 gene was transfected into acinar cells using Lipofectamine 2000 Transfection Reagent (11668500, Thermo Fisher Scientific, USA), with the empty vector used as a negative control (NC). Briefly, after being digested with trypsin (C0205, Beyotime Biotechnology, China), cells were seeded in a 24-well plate at 1 × 10^5^ cells/well and incubated until 70–90% fusion. Lipofectamine 2000 (2.0 *µ*L, at room temperature for 5 min) and DNA (0.8 *µ*g) were diluted in 50 *µ*L Opti-MEM I Reduced Serum Medium without serum (31985062, Thermo Fisher Scientific, USA). Then, the diluted DNA was mixed well with the dilute Lipofectamine 2000 and cultured for 20 min at room temperature, subsequent to which the 100 *µ*L complexes were added into each well and mixed completely by a rocking plate back and forth. Cells were incubated for 48 h in a CO_2_ incubator at 37°C.

### 2.12. Western Blot

Total protein (tissues were cut into small fragments beforehand) was isolated using radioimmunoprecipitation assay (RIPA) buffer (R0020, Beijing Solarbio Science & Technology Co., Ltd., China) and centrifuged at 12000 rpm for 10 min at 4°C. With supernatant harvested, total protein concentration was measured through BCA Protein Assay Kit (PC0020, Beijing Solarbio Science & Technology Co., Ltd., China). Equal amounts of protein (45 *µ*g) and ColorMixed Protein Marker (11–180 kDa) (5 *µ*L; PR1910, Beijing Solarbio Science & Technology Co., Ltd., China) were separated by 6–10% SDS (P0012A, Beyotime Biotechnology, China)-polyacrylamide gel electrophoresis (SDS-PAGE), subsequent to which protein was transferred to PVDF membranes (88585, Thermo Fisher Scientific, USA) blocked in 5% bovine serum albumin (BSA; ST023, Beyotime Biotechnology, China) blocking buffer for 1 h and then incubated at 4°C with rat antipurinergic receptor P2X ligand-gated ion channel 7 (P2X7R, 1 : 1000; sc-134224, Santa Cruz Biotechnology, Dallas, Texas, USA), rabbit anti-NLRP3 (1 : 1000; ab263899, Abcam, Cambridge, MA, USA), rabbit anti-caspase 1 (1 : 1000; ab138483, Abcam, USA), rabbit anti-aquaporin (AQP) 5 (1 : 10000; ab78486, Abcam, USA), rabbit anti-AQP4 (1 : 1000; ab46182, Abcam, USA), rabbit anti-IL-1*β* (1 : 1000; #12426, Cell Signaling Technology, Danvers, MA, USA), rabbit anti-Bax (1 : 2000; ab182733, Abcam, USA), Bcl-2 (1 : 2000; ab182858, Abcam, USA), and mouse anti-GAPDH (1 : 10000; ab8245, Abcam, USA) overnight. Subsequently, membranes were rinsed 4 times with TBST and incubated with corresponding secondary antibodies conjugated to anti-Rat IgG H&L (1 : 5000; ab6734, Abcam, USA), anti-mouse IgG H&L (1 : 5000; ab6728, Abcam, USA), and anti-rabbit IgG H&L (1 : 5000; ab6721, Abcam, USA) for 1 h at room temperature and washed 5 times with TBST for 5 min. Electrochemiluminescence (ECL) Western Blotting Substrate (PE0010, Beijing Solarbio Science & Technology Co., Ltd., China) was utilized to visualize protein through iBright FL1500 Imaging System (Thermo Fisher Scientific, USA). The consequence was analyzed by ImageJ software, version 1.48 (National Institutes of Health, Bethesda, MD, USA).

### 2.13. Statistical Analysis

GraphPad Prism 8.0 (GraphPad Software Inc., San Diego, CA, USA) was adopted for statistical analysis. Data were presented as the means ± standard deviation. All experiments were carried out three times at least. Multiple groups were compared by one-way ANOVA with Tukey's post hoc test. *p* < 0.05 was considered to have a statistically significant difference.

## 3. Results

### 3.1. Ruscogenin Ameliorated the SFR and Submandibular Gland Inflammation of NOD/ShiLtJ Mice

Figure 1(a) shows the chemical structure of Ruscogenin. The SFR did not differ among each group in the early stage. From week 11 to 20, it was viewed that the SFR gradually reduced in NOD/ShiLtJ and vehicle groups (Figure 1(b)), whereas the SFR of mice treated with Ruscogenin did not decrease in comparison with mice treated with vehicle (Figure 1(b), *p* < 0.05), which indicated that Ruscogenin could restore the SS-like symptom. Through histological analysis of submandibular gland, we discovered that both NOD/ShiLtJ and vehicle groups exhibited great infiltration of lymphocytes as well as more inflammation focuses with large area (Figure 1(c)). But the treatment of 0.3 mg/kg Ruscogenin decreased lymphocyte infiltration, the area, and a number of inflammation focuses, with 1 mg/kg Ruscogenin further enhancing that reduction (Figure 1(c)). Similarly, no significant difference in IL-6, IL-17, TNF-*α,* and IL-1*β* mRNA expression was presented in NOD/ShiLtJ and vehicle groups (Figure 1(d)), whereas IL-6, IL-17, TNF-*α,* and IL-1*β* mRNA expression in submandibular gland tissues prominently decreased in the Ruscogenin 0.3 group and the Ruscogenin 1 group when compared to the vehicle group, as the effect of 1 mg/kg Ruscogenin was better than 0.3 mg/kg Ruscogenin (Figure 1(d), *p* < 0.01). Those findings suggested that Ruscogenin improved the SFR and submandibular gland inflammation in a dose-dependent manner.

### 3.2. Ruscogenin Promoted the AQP5 and AQP4 Expression but Suppressed Inflammation-Related Factors in Submandibular Gland Tissues of NOD/ShiLtJ Mice

Through western blot, the AQP5, AQP4, P2X7R, NLRP3, caspase 1, and IL-1*β* protein levels did not differ between the NOD/ShiLtJ and vehicle groups (Figure 2(a)-2(d)). But in contrast with mice treated with vehicle, mice treated with Ruscogenin increased AQP5 and AQP4 protein expression but decreased P2X7R, NLRP3, caspase 1, and IL-1*β* levels; moreover, the effect of the 1 mg/kg Ruscogenin group was better than the 0.3 mg/kg Ruscogenin group (Figure 2(a)–2(d), *p* < 0.05).

### 3.3. Ruscogenin Inhibited the Apoptosis of Acinar Cells in NOD/ShiLtJ Mice and Reversed TNF-*α*-Induced Apoptosis and Inflammation of Acinar Cells

When compared to normal mice (BALB/c), apoptosis of acinar cells in NOD/ShiLtJ mice obviously elevated, whereas the treatment of 1 mg/kg Ruscogenin notably decreased the acinar cell apoptosis of NOD/ShiLtJ mice (Figure 3(a)). To explore the function of Ruscogenin on TNF-*α*-induced acinar cell injury, the acinar cells were cultured with Ruscogenin at different doses (0.1, 1, and 10 *µ*M) prior to exposure to TNF-*α*. The consequence of flow cytometry assay showed a marked rise in the apoptosis rate in cells treated with TNF-*α* (Figures 3(b) and 3(c), *p* < 0.001), while the treatment of Ruscogenin decreased cell apoptosis induced by TNF-*α* as the concentration of Ruscogenin increased (Figures 3(b) and 3(c), *p* < 0.01). Furthermore, cells in the TNF-*α* group exhibited lower AQP5 and AQP4 protein levels with higher NLRP3, caspase 1, and IL-1*β* expression than the control group (Figures 3(d)–3(g), *p* < 0.001). Nevertheless, with the dose of Ruscogenin elevated, cells with cotreatment of TNF-*α* and Ruscogenin gradually elevated AQP5 and AQP4 levels and reduced NLRP3, caspase 1, and IL-1*β* expression in comparison with cells treated with TNF-*α* alone (Figures 3(d)–3(g), *p* < 0.05). Those data implied that Ruscogenin was able to protect acinar cells against TNF-*α*-induced injury.

### 3.4. NLRP3 Reversed the Repressive Effect of Ruscogenin on TNF-*α*-Induced Inflammation and Apoptosis of Acinar Cells

In contrast to the NC group, cells transfected with NLRP3 overexpression plasmid presented a higher NLRP3 protein expression (Figures 4(a) and 4(b), *p* < 0.001), which implicated that transfection succeeded. The result of western blot presented that TNF-*α* treatment increased NLRP3, caspase 1, IL-1*β,* and Bax expression and reduced the Bcl-2 level, while Ruscogenin decreased the TNF-*α*-induced rise of NLRP3, caspase 1, IL-1*β,* and Bax levels and elevated TNF-*α*-induced Bcl-2 downregulation, with NLRP3, caspase 1, IL-1*β,* and Bax protein levels of the TNF-*α*+Ruscogenin 10+NLRP3 group higher than the TNF-*α*+Ruscogenin 10 group, whereas the expression of Bcl-2 in the TNF-*α*+Ruscogenin 10+NLRP3 group is lower than that of the TNF-*α*+Ruscogenin 10 group (Figures 4(c)–4(f), *p* < 0.05), revealing that Ruscogenin might attenuate TNF-*α*-induced inflammation and apoptosis through the inhibition of NLRP3 inflammasome.

## 4. Discussion

SS is an autoimmune disease predominantly affecting women, with major clinical characterizations comprising dry eyes and dry mouth [2, 26]. Ruscogenin is an active component of Ophiopogon japonicas, which exerts various pharmacological properties including anti-inflammatory [23]. However, the functions of Ruscogenin on SS still remain unclear.

We firstly experimented in vivo through establishing animal models of SS with the treatment of Ruscogenin to explore the role of Ruscogenin in SS. In agreement with the research studies about the effect of MDG-1 and green tea polyphenols, as well as AT-RvD1 in SS [12, 16, 27], our study discovered that Ruscogenin recovered the SFR of mice and repressed lymphocytic infiltration and inflammation of submandibular glands, as higher dose of Ruscogenin exhibited better efficacy, which validated the protective role of Ruscogenin against SS. IL-6, IL-17, TNF-*α,* and IL-1*β* are crucial pro-inflammatory cytokines triggering intense inflammatory reaction, whose upregulation has been reported to associate with the pathogenesis of SS [28, 29]. Former studies have shown several promising strategies that can attenuate SS via suppressing inflammation, and Ruscogenin has been proven to restrain inflammation in cerebral ischemic injury, acute lung injury, and blood-brain barrier dysfunction induced by cerebral ischemia [2, 12, 22, 23, 29–33]. Similarly, during our experiments, we observed that Ruscogenin prominently inhibited those inflammation-related factors in NOD/ShiLtJ mice with the increasing concentration of Ruscogenin, implying that Ruscogenin might restore SS through the inhibition of inflammation via the downregulation of pro-inflammatory cytokines in a dose-dependent manner.

Belonging to the AQP family, which is a group of specific water channels allowing the water to move in and out of cells to respond to osmotic/hydrostatic pressure gradients, AQP5 and AQP4 play a key part in forming tears and saliva. AQP5 is located in apical acinar and ductal cells in the lacrimal glands but apically at the membranes of acinar cells in salivary glands, which is believed to provoke the water outflow into the acinar lumen. As for AQP4, it is located laterally in acinar cells of the lacrimal glands, whereas in salivary glands, it is located basolateral membranes of acinar cells [34]. Previous reports have revealed a low expression as well as a disorder of AQP5 and AQP4 in SS animal models and SS patients. And the mutant of AQP5 is confirmed to be correlative with the decrease in the secretion of the salivary gland [2, 25, 34]. It has been reported that mesenchymal stem cells extract-based treatment could improve SS-associated symptoms through upregulation of AQP5 and AQP4 [2]. Consistent with the finding, we also found that Ruscogenin advanced AQP5 and AQP4 levels in NOD/ShiLtJ mice, implying the alleviating potential of Ruscogenin in SS through upregulation of AQP5 and AQP4.

As a vital element in inflammatory responses, the NLRP3 inflammasome, which is a multiprotein complex containing NLRP3 and caspase 1, participates in a variety of diseases including SS [11, 35]. Besides, the involvement of NLRP3 inflammasome has also been confirmed in the effects of Ruscogenin on cerebral ischemia-induced dysfunction of blood-brain barrier [23]. Thus, it could be presumed that the protective role of Ruscogenin in SS might partially attribute to its regulation on NLRP3 inflammasome. To address that, western blot was performed after the treatment of Ruscogenin to evaluate protein levels of factors related to NLRP3 inflammasome. P2X7R is taken as a pivotal receptor in inflammation, whose activation positively connects with the maturation and release of pro-inflammatory molecules like IL-1*β*. In addition, P2X7R is verified to cause inflammatory reactions and exacerbate the prognosis through strongly activating NLRP3 inflammasome [36–39]. Similar to the study about Ruscogenin in blood-brain barrier dysfunction [23], our research viewed that Ruscogenin repressed P2X7R, NLRP3, caspase 1, and IL-1*β* expression in SS mice models in a dose-dependent manner, which implicated that the protective effect of Ruscogenin against SS might be associated with NLRP3 inflammasome.

Secondly, acinar cells were isolated to further investigate the role of Ruscogenin in cells. Through the AO/PI staining assay, it was discovered that Ruscogenin suppressed the elevating apoptosis of acinar cells in NOD/ShiLtJ mice, revealing that perhaps Ruscogenin promoted the preservation of acinar cells. In order to validate whether Ruscogenin could protect acinar cells from inflammation, cells were treated with TNF-*α* to construct a model of cell injury due to the fact that TNF-*α* is capable of inducing cytotoxicity in various kinds of cells [27]. The result of the flow cytometry assay and Western blot presented that TNF-*α* advanced cell apoptosis and pro-inflammatory cytokines while inhibiting AQPs. The similar consequence has been acquired in previous works about the effect of TNF-*α* [13, 25, 40–42]. Those data showed a successful establishment of TNF-*α-*induced cell injury model. MDG-1 has been proved to repress cell apoptosis and inflammation induced by H2O2 [31], in consistent with which, our experiments observed that Ruscogenin reversed those functions of TNF-*α* above in a dose-dependent manner, implying that Ruscogenin indeed protected acinar cells from cell injury via the inhibition of inflammation.

To probe into the specific mechanism of Ruscogenin against SS, NLRP3 overexpression plasmid was transfected into acinar cells, with western blot testing transfection efficiency. Consequently, we found the inhibitory effect of Ruscogenin on TNF-*α-*induced upregulation of NLRP3 inflammasome-related as well as pro-apoptotic (Bax [43]) molecules and downregulation of anti-apoptotic factor (Bcl-2 [43]) were reversed by NLRP3 overexpression plasmid, which suggested that Ruscogenin defended against inflammation and apoptosis in acinar cells via negatively mediating NLRP3 inflammasome. Moreover, in an in vivo experiment, we found that the ameliorate effect of 1 mg/kg Ruscogenin on the NOD/ShiLtJ mice was better than that of 0.3 mg/kg Ruscogenin; in an in vitro experiment, the effect of 10 *µ*M Ruscogenin on the TNF-*α*-induced acinar cells was better than that of 0.1 and 1 *µ*M Ruscogenin.

## 5. Conclusion

As a conclusion, the research clarified a positive role of Ruscogenin against SS and demonstrated that Ruscogenin ameliorated SS by inhibiting NLRP3 inflammasome activation through experiments in vivo and in vitro, providing an innovative and potential drug for SS treatment. But more studies and clinical trials are necessary for further determination of the Ruscogenin's efficacy on SS. In the future research, we will continue to emphasize on more targets of Ruscogenin as well as their mechanisms of action to improve SS management.

## Figures and Tables

**Figure 1:** Ruscogenin ameliorated the SFR and submandibular gland inflammation of NOD/ShiLtJ mice. (a) The chemical structure of Ruscogenin. (b) SFR was calculated using female mice treated with vehicle (sterile PBS) and Ruscogenin (0.3, 1 mg/kg) at weeks 11, 13, 15, 17, and 20. (c) Histological analysis of the submandibular glands in mice treated with vehicle and Ruscogenin (at 20 weeks of age) was conducted by hematoxylin-eosin staining assay. (d) Relative mRNA expression levels of IL-6, IL-17, TNF-*α,* and IL-1*β* in submandibular glands were detected through quantitative reverse transcription-polymerase chain reaction. GAPDH is a loading control. ^*∗*^*p* < 0.05, ^*∗∗*^*p* < 0.01, ^*∗∗∗*^*p* < 0.001 vs. vehicle group. All experiments were repeated independently at least three times. Data were performed as the means ± standard deviation. SFR: salivary flow rate; PBS, phosphate buffer saline; IL: interleukin; TNF: tumor necrosis factor; qRT-PCR: quantitative reverse transcription-polymerase chain reaction; GAPDH: glyceraldehyde-3-phosphate dehydrogenase.

**Figure 2:** Ruscogenin promoted the AQP5 and AQP4 expression while suppressed inflammation-related factors expression in submandibular gland tissues of NOD/ShiLtJ mice. (a and b) Representative images of protein bands (a) and relative protein expression of AQP5 and AQP4 (b) in submandibular gland tissues was tested by western blot after treatment of vehicle and Ruscogenin. GAPDH is a loading control. (c and d) Representative images of protein bands (c) and relative protein expression of P2X7R, NLRP3, caspase 1, and IL-1*β* (d) in submandibular gland tissues was assessed by western blot after treatment of vehicle and Ruscogenin. GAPDH is a loading control. ^*∗*^*p* < 0.05, ^*∗∗*^*p* < 0.01, ^*∗∗∗*^*p* < 0.001 vs. vehicle group. All experiments were repeated independently at least three times. Data were performed as the means ± standard deviation. AQP: aquaporin; GAPDH: glyceraldehyde-3-phosphate dehydrogenase; P2X7R: purinergic receptor P2X ligand-gated ion channel 7; NLRP3: nucleotide binding oligomerization domain-like receptor 3; IL: interleukin.

**Figure 3:** Ruscogenin inhibited the apoptosis of acinar cells in NOD/ShiLtJ mice and reversed TNF-*α*-induced apoptosis and inflammation of acinar cells. (a) Representative pictures of acinar cell apoptosis during AO/PI staining assay after the treatment of Ruscogenin. (b and c) Representative images of cell apoptosis (b) and apoptosis rates (c) were evaluated through flow cytometry assay after the treatment of TNF-*α* and Ruscogenin. (d and e) Representative images of protein bands (d) and relative protein expression of AQP5 and AQP4 (e) in acinar cells was tested by western blot after the treatment of TNF-*α* and Ruscogenin. GAPDH is a loading control. (f and g) Representative images of protein bands (f) and relative protein expression of NLRP3, caspase 1, and IL-1*β* (g) in acinar cells was assessed by western blot after the treatment of TNF-*α* and Ruscogenin. GAPDH is a loading control. ^*∗∗∗*^*p* < 0.001 vs. control group; ^∧^*p* < 0.05, ^∧∧^*p* < 0.01, ^∧∧∧^*p* < 0.001 vs. TNF-*α* group. All experiments were repeated independently at least three times. Data were performed as the means ± standard deviation. TNF: tumor necrosis factor; AO/PI: acridine orange and propidium iodide; AQP: aquaporin; GAPDH: glyceraldehyde-3-phosphate dehydrogenase; NLRP3: nucleotide binding oligomerization domain-like receptor 3; IL: interleukin.

**Figure 4:** NLRP3 reversed the repressive effect of Ruscogenin on TNF-*α*-induced inflammation and apoptosis of acinar cells. (a and b) Representative images of protein bands (a) and relative protein expression of NLRP3 in acinar cells was tested by western blot after the transfection of NLRP3 overexpression plasmid. GAPDH is a loading control. (c and d) Representative images of protein bands (c) and relative protein expression of NLRP3, caspase 1, and IL-1*β* (d) in acinar cells was assessed by western blot after the treatment of TNF-*α* and Ruscogenin as well as transfection of NLRP3 overexpression plasmid. GAPDH is a loading control. (e and f) Representative images of protein bands (e) and relative protein expression of Bax and Bcl-2 (f) in acinar cells was assessed by western blot after the treatment of TNF-*α* and Ruscogenin as well as transfection of NLRP3 overexpression plasmid. GAPDH is a loading control. ^†††^*p* < 0.001 vs. NC group; ^*∗∗∗*^*p* < 0.001 vs. Control group; ^∧∧∧^*p* < 0.001 vs. TNF-*α* group; ^#^*p* < 0.05, ^##^*p* < 0.01, ^###^*p* < 0.001 vs. TNF-*α*+Ruscogenin 10 group. All experiments were repeated independently at least three times. Data were performed as the means ± standard deviation. NLRP3: nucleotide binding oligomerization domain-like receptor 3; TNF: tumor necrosis factor; GAPDH: glyceraldehyde-3-phosphate dehydrogenase; IL: interleukin; NC: negative control for NLRP3 overexpression plasmid.

**Table 1:** Primer sequences used for quantitative reverse transcription-polymerase chain reaction (qRT-PCR).

Target gene	Primers, 5'-3'
IL-6	
(Forward)	TCTATACCACTTCACAAGTCGGA
(Reverse)	GAATTGCCATTGCACAACTCTTT
IL-17	
(Forward)	TCTCCACCGCAATGAAGACC
(Reverse)	CACACCCACCAGCATCTTCT
TNF-*α*	
(Forward)	CCTGTAGCCCACGTCGTAG
(Reverse)	GGGAGTAGACAAGGTACAACCC
IL-1*β*	
(Forward)	GCACTACAGGCTCCGAGATGAAC
(Reverse)	TTGTCGTTGCTTGGTTCTCCTTGT
GAPDH	
(Forward)	TGACCTCAACTACATGGTCTACA
(Reverse)	CTTCCCATTCTCGGCCTTG

## Data Availability

The analyzed datasets generated during the study are available from the corresponding author on reasonable request.
